# Effect of Intervention of Probiotics in Advance on Treg/Th17 in Premature Mice

This article has been retracted.

**DOI:** 10.1155/2022/6131069

**Published:** 2022-07-30

**Authors:** Mengmeng Liu, Juanjuan Mao, Shifa Zhang

**Affiliations:** Department of Pediatrics, Yijishan Hospital, Wannan Medical College, Wuhu, 241001 Anhui, China

## Abstract

To preliminarily understand the differentiation characteristics of regulatory T cells (Tregs) and Th17 at a different time in preterm mice, the impacts of probiotics on immune function progression, as well as the correlation of probiotics with Tregs and Th17. On embryonic day 18 of gestation, a mouse model of preterm birth was built using mifepristone (RU486). Following IPI of RU486, newborn mice were randomized to probiotics or NS gavage administration. Full-term newborn mice were given the same dose of NS gavage administration. Phenotypic analysis of peripheral immune cell frequency was performed using flow cytometry. Cytokine measurements were phenotyped by enzyme-linked immunosorbent assays. On the 14th and 21st days after birth, the highest and lowest expressions of Foxp3, the Treg transcription factor, were observed in full-term mice and premature mice by NS gavage administration, respectively, while the opposite trend was found in the Th17 transcription factor IL-17.IL-2, IL-6, and TGF-*β* rose with age but showed different trends among the three groups. IL-2 is the highest in full-term mice and the lowest in premature mice. IL-6 and TGF-*β* is the lowest in full-term mice and the highest in premature mice. Probiotics are beneficial to the development and maturation of the immune system, which may play a role in regulating the ratio of Treg/Th17. Probiotic preintervention can effectively promote the differentiation of Treg and inhibit the differentiation of Th17 in premature mice. Its mechanism of action may play a biological role by regulating cytokine (IL-2, IL-6, and TGF-*β*) secretions.

## 1. Introduction

The preterm birth (PTB) rate increased to 10.02% for the fourth consecutive year, as indicated by U.S. Births 2018 [1]. According to the World Health Organization (WHO), PTB refers to any birth that occurs before 37 completed weeks of gestation or delivery with a period < 259 days since the mother's last menstrual period (LMP) [2]. Approximately 85% of these births are moderate (32-33 weeks) to late preterm babies (34-36 weeks), with 10% and 5% being very preterm (28-31 weeks) and extremely preterm (<28 weeks) babies, respectively. For neonates, PTB is a risk factor that impacts their growth and health well into adult life. Also, preterm babies face increased mortality and morbidity outcomes than term infants. With the development and progress of medical technology, the survival rate of preterm infants has been greatly improved and the quality of life in adulthood has been improved. The latest study suggested increased feeding difficulties and risks of visual and hearing problems, as well as neonatal septicemia, respiratory distress syndrome, neurological disorders, bronchial-pulmonary dysplasia, and necrotic enterocolitis as the short-term complications of prematurity [3, 4].

The complications of premature infants are mostly related to the incomplete immune system. It has been well demonstrated that regulatory T cells (Tregs), a subpopulation of CD4^+^T cells, are capable of modulating and suppressing the immune system [5] and are vital in autoimmunity (AI). During infection, they can work both for and against the host, controlling excessive host immunoreaction. Advances have been made in the cellular biology of Tregs along with the discovery of forkhead box p3 (Foxp3), a gene encoded by the X chromosome. Subsequent studies showed that for mature Tregs, sustained Foxp3 expression is a must for their maintenance and suppressive action [6].CD4+ T helper (Th) cells are pivotal in tissue destruction in a wide spectrum of inflammatory and autoimmune diseases (AIDs). Interleukin- (IL-) 17-producing Th (Th17) cells belong to an inflammatory Th subpopulation among all Th subpopulations, which can give rise to chronic tissue inflammation and even organ failure. Hence, a better understanding of Th17 cell differentiation and pathogenic functions carries huge implications for developing novel immunotherapies for inflammatory diseases associated with Th17 [7]. It is considered that Th17 cells are the primary driver of etiopathogenesis, triggering inflammation via activating multiple cell types (macrophages, DCs, and synoviocytes) within the inflamed joint. There is growing evidence showing that Th17/Treg balance is the basis of the nosogenesis leading to AIDs [8, 9].

The differentiation of various CD4+ T cell subpopulations from naïve CD4+ T cells is accurately controlled by multifaceted interactions of cytokines (CKs) and microRNAs that are responsible for multifaceted subset-specific transcription factors, to ensure a balance among them [10, 11]. Therefore, it has great clinical implications for exploring factors participating in naive T cell differentiation to CD4+ T cell subpopulations and optimizing the methods for fine-tuning the specific responses of subpopulations. Foxp3 interferes with the growth and functioning of CD4+CD25+ Treg cells, which exert vital effects on AI, anti-infection immunity, tumor immunity, and transplantation tolerance via generating anti-inflammatory CKs like transforming growth factor TGF-*β* and IL-10. Naïve CD4+ T cells can be differentiated into Tregs via TGF-*β* intervention, whereas cotreatment with TGF-*β*+ IL-6 promotes differentiation into Th17 cells. The naïve CD4+ T is the shared precursor of both Th17 and Treg cells, and a common TGF-*β* signal is required for their initial differentiation. But the cells that are terminally differentiated have the opposite function: Th17 can enhance AI and inflammation, whereas Treg can maintain immunologic homeostasis. So, it is critical to clarify the mechanisms underlying the Th17-Treg balance to better understand AI and tolerance [12].

Herein, we probed into the role played by probiotics in premature mice and the balance between Tregs/Th17. Its mechanism of action may play a biological role by regulating CK (IL-2, IL-6, and TGF-*β*) secretions.

## 2. Data and Methods

### 2.1. Animals

8-10-week-old BALB/c mice with a weight of 18 to 22 g were supplied by the Animal Center of Nanjing Qinglong Mountain (Nanjing, China) and raised with food and water ad libitum under the following specific pathogen-free conditions during the entire study process: 12 h light-dark cycle, 21 ± 2°C, and humidity: 45 ± 10%. After mating, timed fertile mice were obtained for research. To build a PTB model, fertile mice were randomized to receive mifepristone (RU486), a progesterone receptor antagonist. Intraperitoneal injection (IPI) of 1 mg RU486 in normal solution (NS) was carried out on gestation day 18. After IPI of RU486, premature animals were stochastically selected for gavage treatment with either probiotics or NS for 7 days. The 3 treatment groups, namely, RU486+probiotics (group A), RU486+NS (group B), and NS+NS (group C), were compared in this study according to the study protocol. On the day 14th and 21st, 15 newborn mice from each treatment group were randomly selected for these experiments. The mice conducted all studies according to the guidelines from the National Institutes of Health and People's Republic of China legislation regarding laboratory animal use and care.

### 2.2. Flow Cytometry

To dye IL-17A, an intracellular CK, mouse peripheral blood was immersed in a 1x cell-stimulating cocktail comprising protein transport inhibitors(500xX) for 6 h. After harvesting the cultures, they were subjected to immobilization and permeabilization using IC fixation buffer (cat. no. 00-822) and permeabilization buffer (cat. no. 00-8333, Thermo Fisher Scientific, Shanghai, China), respectively. This was followed by cell staining with Anti-Mouse CD4 PE-CY-5 (cat. no. 553050, BD, New Jersey, USA) and Anti-Mouse CD25 BB515 (BD, cat. no. 564424) (30 min, 2-8°C). The cells were centrifuged (350 × g, 5 min) after one rinsing with a staining buffer (2 ml). Then, intracellular staining for Foxp3 was carried out. After completing cell surface staining, the residual stain buffer was removed and the cell mass was briefly loosened by vortexing. Then, came the addition of Fix/Perm Buffer working solution to each tube for cell mass resuspension by vortexing for 3 secs. or so. Thereafter, the specimens were treated with light-tight cultivation (2-8°C, 40-50 min). Finally, stained cells with Anti-Mouse IL-17A PE (BD, cat. no. 559502) and ANTI-M/R Fox3 PE-Cy-7(BD, cat. no. 25-5773-82).

### 2.3. FACS Antibodies

Antibodies for FACS included PBB515 Rat Anti-Mouse CD25 (BD, cat. no.564424), PE-Cy-5 Rat Anti-Mouse CD4 (BD, cat. no.553050), PE-Cy-7 ANTI-M/R Foxp3 FJK-16S (BD, cat. no.25-5773-82), and PE Rat Anti-Mouse IL-17A (BD, cat. no.559502).

### 2.4. Enzyme-Linked Immunosorbent Assays (ELISAs)

On days 14 and 21, blood specimens from all groups were collected. The quantification of CK (IL-2, IL-6, and TGF-*β*) protein levels was made by the commercial ELISA kits following the manufacturer's instructions (Shanghai Elisa Biotech Co., Ltd., Shanghai, China). Briefly, serum specimens after dilution were placed into the wells of purified anti-IL-2, IL-6, and TGF-*β* first polyclonal antibody-coated 96-well plates, after which the specimens were washed and incubated as indicated in the manual. A microplate reader was utilized to read the absorbance_450nm_, and the concentrations were denoted by pg/ml.

### 2.5. Statistical Processing

The significance level was judged by appropriate statistical analysis based on whether the data were in normal distribution and the number of test groups available for comparison. LSD test was performed to determine whether there was any significance in multigroup comparisons. GraphPad Prism *v*8.2.1 (GraphPad Software, San Diego, USA) was adopted. *P* < 0.05 was the threshold of significance.

## 3. Results

### 3.1. Proportions of Peripheral T Cells

We first investigated the differences in the frequencies of T cells in mouse blood sample. As shown in Figures 1(a) and 1(b), CD4+ T cells were gated in the lymphocyte population and the CD4+CD25+ high fraction was determined by a fluorescence intensity. Meanwhile, Th17 cells (IL-17A+CD4+) and Foxp3 were expressed in CD4+ T cells.

### 3.2. Tregs

Not only on the 14th but also 21st, the expression of Foxp3 was elevated in group A versus group B but was lower when compared to group C (*P* < 0.05). Nevertheless, the percentage of Foxp3 in the three groups increased in the overall trend, as shown in Figure 2.

### 3.3. Th17

The mean Th17 level was the highest in group B, followed in descending order by groups A and C (*P* < 0.05) obviously, a significant difference was observed among the three groups, as shown in Figure 3.

### 3.4. Il-2

On the 14th and 21st day after birth, the concentration of IL-2 was the highest in group C, followed in descending order by groups A and B (*P* < 0.05). Nevertheless, IL-2 in the three groups increased in the overall trend, as shown in Figure 4.

### 3.5. Il-6

The mean IL-6 value was the lowest in group C and highest in group B, with that in group A in between (*P* < 0.05). Obviously, a significant difference was observed among the three groups, as shown in Figure 5.

### 3.6. TGF-*β*

The mean TGF-*β* value was the lowest in group C, followed in ascending order by groups A and B (*P* < 0.05); obviously, a significant difference was observed among the three groups, as shown in Figure 6.

### 3.7. Probiotics Facilitated Treg Differentiation while Suppressing Th17 Differentiation

Tregs and Th17 cells isolated from peripheral blood were analyzed by flow cytometry. Fox P3 was higher in group A versus group B but was lower when compared to group C. The result of IL-17 expression showed an inverse trend. Thus, IL-17, a Th17 cell-related CK declined; while Foxp3, a Treg cell-related CK elevated, demonstrating that it can validly suppress inflammation and may also modulate Th17/Treg equilibrium, as shown in Figures 2 and 3.

### 3.8. Probiotics May Exert Their Effects by Regulating CKs (IL-2, IL-6, and TGF-*β*)

IL-2 in group A was increased noticeably versus the control group (B), although still lower than in group C. IL-6 and TGF-*β* were highest in group B while lowest in group C. Thus, it was indicated that IL-2 was beneficial for Treg differentiation but IL-6 and TGF-*β* were beneficial for Th17, as shown in Figures 4–6.

## 4. Discussion

PTB is a major public health issue, which predisposes preterm babies to innate and adaptive immune response (IR) deficiency featured with reduced IgG, opsonic action, and phagocytosis. PTB bears responsibility for nearly 1,000,000 deaths in children aged under five. Ascending congenital infection and fetal inflammation are believed to be the main inducements of PTB, though the exact nosogenesis remains to be clarified [13]. A newborn's immune system is known to be not mature enough after delivery, with its adaptive IR (specificity and memory) continuing to develop into early childhood [14], which may explain reduced IgG, as well as poor opsonic action and phagocytosis of pathogens as mentioned above. In recent years, probiotics are an immunomodulatory function, which affects the physiological function of the host [15]. Abundant studies have provided evidence of the effectiveness of probiotics in treating AIDs, pathogenic infections, bone immune system, cancer, etc. [16, 17]. By involving in the process of immune regulation, probiotics can create and maintain systemic immunity on the surface of the intestinal mucosa, which can be transformed into enhancing the extensive immunity of the whole body [18].

In this study, we probed into the differentiation characteristics of Tregs and Th17 at different times in preterm mice. The results found that the percentage of Tregs in mice was higher than in the control group by the intervention of probiotics, but the level of Tregs was still lower than in mature mice. Meanwhile, Foxp3, the Treg transcription factor, was found to be the highest and lowest in full-term and premature mice by NS gavage administration, respectively, while an inverse trend was observed in IL-17, a th17 transcription factor. The increase of Tregs' numbers or function may be due to using probiotics, which can regulate the innate IR. Treg cells are of critical importance for maintaining immunologic homeostasis. FoxpP3 functional loss can cause fatal autoimmune autoimmunity diseases, immune disorders, enteropathy, polyendocrinopathy, and X-linked in humans and mice [17]. T cells are crucial and play a vital part in various adaptive IRs. Naïve T helper cells can differentiate into different subsets (Th1, Th2, Treg, and Th17) according to environmental stimuli (antigens, CKs, etc.) during activation. This balance is promoted by probiotics, which further have a huge impact on the anti-inflammatory and pro-inflammatory response in the body. In a report published in 2010, experimental mice with AIDs were treated with two probiotic strains, and enhanced Naïve T cell differentiation into Tregs was observed, which helped to reduce the symptoms of AIDs [19]. On the contrary, it was found that Th17 cells proliferated in mice with suppressed immune conditions after treatment with probiotic strains in a study published in 2016 [20].

Then, we further investigated the underlying mechanism and found that the level of IL-2, IL-6, and TGF-*β* raised with age but showed different trends among the three grows. Among them, the highest IL-2 level was found in full-term mice and the lowest was observed in premature mice while IL-6 and TGF-*β* were the lowest in full-term mice and the highest in premature mice. Based on most in vitro studies, probiotics or their components are considered to affect T-helper type 1 (Th1) or regulate the stimulation of CKs, which more specifically control the Th2 metamorphic phenotype [21]. The immunomodulatory properties of probiotics can be roughly divided into the anti-inflammatory and proinflammatory reactions induced by probiotics. The proinflammatory response induced by probiotics to pathogenic microorganisms may lead to increased secretion of proinflammatory CKs. The anti-inflammatory response caused by probiotics may include the increase of regulatory T cells (Treg) and CKs [22]. There is growing evidence that ≥7 distinct Th subpopulations differentiate as a response to specific CK combinations. For example, iTregs can be induced by TGF-*β* and IL-2, and Th17 by TGF-*β*, IL-21, and IL-6 [10]. In this case, it is suggested that inflammation can be alleviated by probiotics in such a way. Probiotics *B. adolescentis* has been shown to deliver probiotic-mediated adaptive immune regulation to the Treg/Th17 axis via the TRL2/ERK/MAPK/NF-*κ*B axis, stimulating immunosuppressive macrophage polarization and IL-10 secretion [23].

The adaptive IR is an antigen-specific, immune-memory-dependent, and T- and B-cell-dependent response because different patterns of T-cell receptor gene recombination are more specific in identifying invasive substances, thus efficiently promoting T cell activation and antibody synthesis. Tregs are crucial to immunologic homeostasis maintenance. Foxp3 is the key transcription factor for Tregs differentiation and function. Foxp3, the lineage-determining transcription factor for Tregs, is an X-chromosome-encoded member of the Forkhead family [15, 16]. We found that the percentage of Tregs in mice was higher than in the control group by the intervention of probiotics, but the level of Tregs was still lower than in mature mice. It is possible that the increase in Tregs' numbers or function is due to using probiotics, which can regulate the innate IR.

Due to their ability to adjust defense against specific pathogens and the unique CKs and effector functions that mediate tissue inflammation, Th cells are considered a crucial arm of the adaptive immune system. Th17 cells, the latest discovered and the third subpopulation of effector Th cells are effective in host defense against specific pathogens and powerful inducers of tissue inflammation and AI [24]. Besides, the differentiation factors that lead to their production reveal an interesting reciprocal relation with Tregs, which mediate self-tolerance and block tissue inflammation. Th17 can produce mass IL-17A, and TH17-mediated effects are mainly caused by this CK. IL-17A is the prototypic CK among the six members (IL-17A, B, C, D, E, and F) of the IL-17 family [25]. Apart from IL-17A, IL-17F was coproduced by TH17 [26, 27], both of which can induce the secretion of proinflammatory CKs, matrix metalloproteinases, and chemokines from all kinds of tissue and cell types, with shared functions. This study found that the use of probiotics contributed to reduced Th17 compared with the control, thereby reducing IL-17 production. Many studies have confirmed [28, 29], with potent proinflammatory action, that IL-17 induces tissue injury in various AIDs [30].

Th17-Treg balance has become an important element in regulating AI and cancers. Here, TGF-*β* was mainly produced by Tregs while IL-6 by LPS-stimulated monocytes. Combining the other two reports [31, 32], all these data support the role of IL-6 as a critical factor for Th17 differentiation. However, not only IFN-*γ* and IL-4 but also IL-2 (at least early in the differentiation process) can inhibit Th17 differentiation initiation [33]. As to the mechanism, IL-2 downmodulates both gp130 and IL-6Rɑ on conventional T cells, thereby lowering their responses to IL-6 [34].

## 5. Conclusions and Perspectives

Since Th17 cells promote inflammatory responses and Tregs alleviate inflammation in many AIDs, Th17-Treg balance is of great implications for pathogenesis exploration, prognosis assessment, and therapy development.

Collectively, using probiotics as early as possible reduced Th17 but increased Tregs in a mouse PTB model. The immunological function can be ameliorated in a mouse PTB model through probiotics intervention. The modulation may be linked to CD4 T cell differentiation towards the Treg/Th17 equilibrium, which was influenced by CKs IL-2, IL-6, and TGF-*β*.

## Figures and Tables

**Figure 1:** Proportions of peripheral T cells in mouse blood sample ((a) the gating strategy for CD4+ cells in mouse blood sample, (b) representative flow cytometric dot plots of CD4+CD25+ T cells, (c) Representative flow cytometric data of CD4+IL-17A+ T cells, and (d) representative flow cytometric data of CD4 + CD25+Foxp3+ T cells).

**Figure 2:** Foxp3 expression among treatment groups. *P* < 0.05 vs. group C.

**Figure 3:** IL-17 expression. *P* < 0.05 vs. group C.

**Figure 4:** Concentration of IL-2 among treatment groups. *P* < 0.05 vs. group C.

**Figure 5:** Concentration of IL-6 among treatment groups. *P* < 0.05 vs. group C.

**Figure 6:** Concentration of TGF-*β*. *P* < 0.05 vs. group C.

## Data Availability

The labeled dataset used to support the findings of this study are available from the corresponding author upon request.
